# Enhanced Laterality Index: A Novel Measure for Hemispheric Asymmetry

**DOI:** 10.1155/2022/8997108

**Published:** 2022-04-29

**Authors:** Yuwen Li, Zhimin Zhang

**Affiliations:** ^1^School of Instrument Science and Engineering, Southeast University, Nanjing 210000, China; ^2^Science and Technology on Information Systems Engineering Laboratory, The 28th Research Institute of CETC, Nanjing 210000, China

## Abstract

During sleep, the two hemispheres display asymmetries in their activation pattern. Various hemispheric asymmetry measures have been utilized in existing works. Nevertheless, all these measures have one common problem that they would merely take one representative quantity into account when evaluating the functional asymmetry. However, there is a complex series of information exchanges between the two cerebral hemispheres, and only considering one quantity inevitably leads to one-sided or even incorrect conclusions. Consequently, to address the limitation of conventional laterality indices, we propose the so-called enhanced laterality index (ELI), which considers multiple measures of functional asymmetries. Normal sleep and obstructive sleep apnea electroencephalograms (EEGs) from 21 subjects collected in the clinical acquisition system are applied, and two representative quantities are considered simultaneously in this paper. We measure the signal complexity by using fuzzy entropy, and the signal strength is evaluated by calculating EEG energy. The difference of ELI is demonstrated by the comparison with the traditional laterality index (LI) in evaluating the functional asymmetry during sleep.

## 1. Introduction

Hemispheric oscillation of slow-wave activity in the brain during sleep is well manifested in animals, such as birds and cetaceans [1–3], and its research in humans is gradually arousing people's attention recently [4–7]. The asymmetry processing of sensory, affective, and cognitive information is believed to be one of the intriguing properties of human brain function. It is widely accepted that both cerebral hemispheres are in constant communications with each other during all kinds of brain activities [8]. At the same time, the differences between left and right cerebral hemispheres have been reported in existing studies with EEG [9, 10] and fMRI [11], including language, vision, audition, and memory [12].

First of all, a reliable measure that can accurately evaluate the hemispheric asymmetry is needed [13, 14]. In the past, existing works have proposed or applied different kinds of indices to investigate the differences between the two cerebral hemispheres. The most commonly used one is called the laterality index (LI) [15] or asymmetry index in other works [16]. The computation of LI is defined as LI=*λ* · (*Q*_*LH*_ − *Q*_*RH*_)/(*Q*_*LH*_+*Q*_*RH*_), where *Q*_*LH*_ and *Q*_*RH*_ are representative quantities measured for left and right hemispheres, respectively. The parameter *λ* is a scaling factor that defines the range of LI values. The major rational for using LI values to measure hemispheric differences lies in that it facilitates the description of hemispheric asymmetry from functional activation patterns because it is easier to manipulate one value per subject than thousands of voxels. When interpreting LI values and comparing between subjects, there are several factors that need to be taken into consideration including the nature of quantification of left and right hemisphere contributions, the localization of volumes of interest within each hemisphere, the thresholding LI, and so on. At the same time, some modifications to the traditional LI equation have also been proposed. In [15], a modified LI was proposed to solve the problem of negative *Q*_*LH*_ and *Q*_*RH*_ values, while Nagata et al. also presented an alternative way to minimise the influence of the threshold on LI assessment [17].

In addition to LI and its modifications, some other measures have also been proposed or applied in existing publications. Magnitude of squared coherence (MSC) is the modulus of the coherence function measuring the linear correlation in amplitude and phase between two signals. In [18], MSC was applied to C3 and C4 EEG signals in the frequency domain to investigate the asymmetric sleep in human patients, and their work reported an increase of MSC in the delta EEG range during apneic episodes. Besides, the phase lag index (PLI) is a measure of linear and nonlinear interhemispheric phase synchrony, and it is sensitive to phase differences between two EEG signals. Rial et al. reported that the left hemisphere was the dominant during the air flux since the PLI corresponding to the delta band was positive and different from zero. In addition, the index *L* measures the nonlinear synchronization between two signals in their reconstructed state space using the concept of generalized synchronization. The calculation procedure of index *L* refers to [18], and their work reported an obvious increase in index *L* during apneic events. In general, all the three indexes mentioned above show obvious and consistent changes in interhemispheric symmetry depending on the state of the airways during sleep. At the same time, some works related to functional asymmetries of the brain associated with EEG-arousals were also manifested by two other indexes, called interhemispheric asynchrony (IHA) [19] and interhemispheric synchrony index (IHSI) [20]. IHA is computed based on the spectral correlation coefficients over all EEG frequency bands, while IHSI is based on the higher order spectral of IHA time series and principal component analysis [20].

In general, all the abovementioned indexes have been successively applied to demonstrate the functional asymmetries between two cerebral hemispheres during sleep apnea or EEG-arousal in existing publications. However, one common problem that desperately needs to be solved in all the abovementioned indexes is that they merely take only one representative quantity into account when calculating the index. For example, only the power spectrum of 30 seconds of EEG time series was acquired to calculate LI in [21], and only the voxels that survive a fixed threshold within regions of interest of fMRI were counted to calculate LI in [15]. Besides, other examples were also given in [18] that only the correlations between two signals from each hemisphere were considered for MSC, only the relative phase between two signals from each hemisphere was considered for PLI, and only the degree of the interdependence between two signals from each hemisphere was considered for index L. In addition, both IHA and IHSI only considered the spectral correlation coefficients of signals from both hemispheres [19, 20]. However, brain activities involve a complex series of information exchanges between two hemispheres; the conventional LI and its modifications do not account for multiple representative quantities in evaluating hemispheric asymmetry. Consequently, we intend to solve this problem by proposing a more reliable index called the enhanced laterality index (ELI), which could consider more than one representative quantity from both hemispheres. Compared with the existing indexes, ELI would make more reliable conclusions since the information from different quantities would be integrated and analyzed simultaneously. Extensive experiments on normal sleep and obstructive sleep apnea (OSA) EEG data were conducted in this paper to test the effectiveness of ELI.

The remaining sections of this paper are organized as follows: the clinical data acquisition and ELI definition are given in Section 2, the results on the traditional LI and the proposed ELI are presented in Section 3, while discussions and conclusions are given in Sections 4 and 5, respectively.

## 2. Materials and Methods

### 2.1. Clinical Data Acquisition

The clinical data applied in this paper are acquired in the Sleep Medical Centre of Shandong Provincial Hospital, China. Patients suspected of suffering from sleeping problems, including OSA or snoring, are referred to the hospital for a routine overnight diagnostic test known as the polysomnography test (PSG). Patients were monitored by the Respironics Alice 5 PSG Diagnostic Sleep System during overnight sleep. Electrodes were placed in the basic sleep diagnostic montage, pressure and thermal sensors are used for the oral and nasal airflow, and Nonin finger probes are used for blood oxygen saturation.  Table 1 presents the demographic details of the subjects in this study. We include 21 subjects in this study with 9 females and 12 males aged from 18 to 85 years. The corresponding sleep efficiency, apnea-hypopnea index (AHI), sleep arousal, and SpO_2_ (pulse oxygen saturation) for each individual subject are also given.

Sleep efficiency is the percentage of time spent sleeping while in bed. AHI is an index used to indicate the severity of sleep apnea. It is represented by the number of apnea and hypopnea events per hour of sleep. The AHI is calculated by dividing the number of apnea events by the number of hours of sleep. AHI values are categorized as: normal: 0–4; mild sleep apnea: 5–14; moderate sleep apnea: 15–29; severe sleep apnea: 30 or more. Arousal is an abrupt change in the pattern of brain wave activity, as measured by an EEG. Arousal typically represents a shift from deep sleep, which is commonly known as REM sleep, to light sleep, known as NREM sleep, or from sleep to wakefulness. SpO2 is a measurement of the amount of oxygen attached to the haemoglobin cell in the circulatory system. Put simpler, it is the amount of oxygen being carried by the red blood cell in the blood. The normal range of SpO_2_ is around 96%.

In our overnight PSG test, multiple medical signals are carefully monitored simultaneously. To be specific, electrooculogram (EOG), EEG, electromyography (EMG), nasal/oral airflow, respiratory effort, SpO_2_, body positions, body movements, and snore are included in this test for an individual patient. Altogether, a PSG test involves over 24 channels of measurements requiring physical contact with the patient. The recorded PSG data are manually given annotations by sleep technicians according to the American Academy of Sleep Medicine (AASM) [22] so that the sleep stages and REM/NREM status of sleep could be determined. All related sleep diagnosis were made according to the standard diagnostic criteria of the International Classification of Sleep Disorders [23].

Two channels of EEG signals, C3-A2 and C4-A1, recorded with and without OSA occurring are segmented separately for further analysis. Each segment lasts 20 seconds. Since the sampling frequency in the acquisition system is 200 Hz, 4000 data points are included in each segment. Besides, it is necessary to mention that EEG data are recorded from the cortical regions of both hemispheres using electrode positions, C4, C3, A2, A1, based on the standard international 10–20 system of electrode placement [24].  Figure 1 gives typical examples of 20 s epoch C3-A2 and C4-A1 EEG for both normal sleep and OSA segment.

The data studied in this paper were acquired in clinical diagnosis. As a part of the analysis and also one advantage of these PSG data, the event types are also carefully annotated at the exact time positions throughout the whole measurement (see Figure 2). Possible event types such as central apnea, obstructive apnea, hypopnea, leg movement, snore, long RR, heart rate rise, µ-arousal, and PTT drop are annotated for each individual patient. Consequently, the exact signal segments related to specific event types could be easily acquired. This helps to mine data features to the greatest degree for each kind of event.

### 2.2. Enhanced Laterality Index

Generally, in order to recognize the interrelationships between the two brain hemispheres, the most commonly used data analysis index is called the laterality index (LI). In this paper, we propose a novel analysis index called enhanced laterality index (ELI) which could capture multiple kinds of representative quantities measured from left and right hemispheres simultaneously. ELI is defined as follows:

(1) $$\begin{array}{c} \text{ELI}=\sum_{i=1}^{N}\lambda_{i}\cdot \frac{Q_{\text{LH}}^{i}-Q_{\text{RH}}^{i}}{Q_{\text{LH}}^{i}+Q_{\text{RH}}^{i}}\\ =\lambda_{1}\cdot \frac{Q_{\text{LH}}^{1}-Q_{\text{RH}}^{1}}{Q_{\text{LH}}^{2}+Q_{\text{RH}}^{2}}+\lambda_{2}\cdot \frac{Q_{\text{LH}}^{2}-Q_{\text{RH}}^{2}}{Q_{\text{LH}}^{2}+Q_{\text{RH}}^{2}}+\cdots +\lambda_{N}\cdot \frac{Q_{\text{LH}}^{N}-Q_{\text{RH}}^{N}}{Q_{\text{LH}}^{N}+Q_{\text{RH}}^{N}}, \end{array}$$

where

(2) $$\begin{array}{c} \sum_{i=1}^{N}\lambda_{i}=1, \end{array}$$

*Q*_LH_^*i*^ and *Q*_RH_^*i*^ represent the *i*^th^ quantity measured from the left and right hemispheres, respectively, and *λ*_*i*_ is the scaling factor that makes a tradeoff between *N* quantities. Concretely, for a given set of *λ*_*i*_, ELI would vary continuously from 1,   which represents for a pure left hemisphere asymmetry, to –1 that represents for a pure right hemisphere asymmetry. Specifically, when *N*=1, ELI degrades into the traditional LI.

#### 2.2.1. Step A: EEG Data Segmentation and Data Preprocessing

- (A1) According to the event type annotation (see Figure 1), 20 seconds of C3-A2 and C4-A1 EEG data related to normal sleep and OSA are segmented for each subject. Let the digitized EEG data from the left hemisphere of the brain during PSG be *x*_*C*3_^*i*^ and data segmented from the right hemisphere be *x*_*C*4_^*i*^, where *i* represents the number of subject that ranges from 1 to 21 since we include 21 subjects in total in this study.
- (A2) To remove the high frequency artifacts such as the muscle noise and power line interference at 50 Hz, the data acquired in step A1 passes through an 8^th^-order digital Butterworth filter (see Figure 3(a)) with the cutoff frequency *f*=50 Hz to obtain the filtered segments *y*_*C*3_^*i*^ and *y*_*C*4_^*i*^. Typical examples of the spectrum of the original signal and the filtered signal are illustrated in Figure 3(b).
- (A3) The filtered EEG data *y*_*C*3_^*i*^ and *y*_*C*4_^*i*^ are differentiated into frequency bands, delta (*δ*, 1–3 Hz), theta (*θ*, 4–7 Hz), alpha (*α*, 8–13 Hz), and beta (*β*, 14–30 Hz) [25], based on the wavelet transform. Let the resulting spectral magnitude be denoted by *y*_*k*_^*iδ*^, *y*_*k*_^*iθ*^, *y*_*k*_^*iα*^, and *y*_*k*_^*iβ*^ respectively, where *k* represents C3 or C4 channel.  Figure 4 presents the four typical frequency bands, *δ*, *θ*, *α*, and *β*, decomposed from the original recorded EEG.

#### 2.2.2. Step B: Computation of Representative Quantities

In this step, signal complexity and signal strength are considered simultaneously to determine the hemispheric brain asymmetry during normal sleep and OSA:

(i) (*B1) Computation of Fuzzy Entropy*. The detailed physical significance of fuzzy entropy refers to [26–28]. For a decomposed EEG frequency component *y*_*k*_^*ij*^, where *j* denotes *δ*, *θ*, *α*, or *β*, it is segmented into 20 epochs evenly. Each epoch is notated as *y*_*k*_^*ij*^*|*_*l*_, where *l* ranges from 1 to 20, and it lasts 1 second and 200 data points. The fuzzy entropy (FE) of each *y*_*k*_^*ij*^*|*_*l*_ is then computed as follows:
  (3) $$\begin{array}{c} \begin{array}{c} {{\text{FE}}_{k}^{ij}|}_{l}\left(m,n,r\right)=\ln\;\phi^{m}\left({y_{k}^{ij}|}_{l},n,r\right)-\ln\;\phi^{m+1}\left({y_{k}^{ij}|}_{l},n,r\right) \end{array}, \end{array}$$
where *m* is the embedding dimension, *n* is the fuzzy power, *r* is the tolerance threshold [26], and
  (4) $$\begin{array}{c} \phi^{m}\left({y_{k}^{ij}|}_{l},n,r\right)=\frac{1}{N-m+1}\sum_{s=1}^{N-m+1}\left(\frac{1}{N-m}\sum_{t=1,t\neq s}^{N-m+1}\left(\exp\left(-\frac{{\left(d_{st}^{m}\right)}^{n}}{r}\right)\right)\right), \end{array}$$
where *N* = 200 and *d*_*st*_^*m*^ is the maximum distance between two subsequences segmented from *y*_*k*_^*ij*^*|*_*l*_, i.e., ${Y_{k}^{ij}|}_{ls}=\left\{{y_{k}^{ij}|}_{l}\left(s\right),{y_{k}^{ij}|}_{l}\left(s+1\right),\ldots ,{y_{k}^{ij}|}_{l}\left(s+m-1\right)\right\}-\bar{{y_{k}^{ij}|}_{l}}$ and ${Y_{k}^{ij}|}_{lt}=\left\{{y_{k}^{ij}|}_{l}\left(t\right),{y_{k}^{ij}|}_{l}\left(t+1\right),\ldots ,{y_{k}^{ij}|}_{l}\left(t+m-1\right)\right\}-\bar{{y_{k}^{ij}|}_{l}}$, in which $\bar{{y_{k}^{ij}|}_{l}}$ represents the mean value of *y*_*k*_^*ij*^*|*_*l*_. Finally, the average fuzzy entropy for the entire sequence *y*_*k*_^*ij*^ could be computed as follows:
  (5) $$\begin{array}{c} \begin{array}{c} {\text{FE}}_{k}^{ij}=\frac{1}{20}\sum_{l=1}^{20}{{\text{FE}}_{k}^{ij}|}_{l}\left(m,n,r\right) \end{array}. \end{array}$$
(ii) *(B2) Computation of Signal Strength*. Similarly, *y*_*k*_^*ij*^*|*_*l*_ is firstly acquired, and the energy of this signal segment is computed as follows:
  (6) $$\begin{array}{c} \begin{array}{c} {E_{k}^{ij}|}_{l}=\sum_{s=1}^{N}{\left({y_{k}^{ij}|}_{l}\left(s\right)\right)}^{2} \end{array}. \end{array}$$
Consequently, the average energy of the entire sequence *y*_*k*_^*ij*^ could be computed by the following equation:
  (7) $$\begin{array}{c} \begin{array}{c} E_{k}^{ij}=\frac{1}{20}\sum_{l=1}^{20}{E_{k}^{ij}|}_{l} \end{array}. \end{array}$$

#### 2.2.3. Step C: Computation of ELI

(i) (C1) Computation of LI only considering signal complexity. Since the fuzzy entropy of two channels (C3 and C4) and four frequency bands (*δ*, *θ*, *α*, or *β*) of each subject could be computed using (5) in step B1, then LI based on the signal complexity could be computed as follows:
  (8) $$\begin{array}{c} \begin{array}{c} {{\text{LI}}_{\text{FE}}|}_{ij}=\frac{{\text{FE}}_{C3}^{ij}-{\text{FE}}_{C4}^{ij}}{{\text{FE}}_{C3}^{ij}+{\text{FE}}_{C4}^{ij}} \end{array}. \end{array}$$
(ii) (C2) Computation of LI only considering signal strength. Similarly to step C1, the average energy of two channels (C3 and C4) and four frequency bands (*δ*, *θ*, *α*, or *β*) of each subject could be computed using (7) in step B2, then LI based on signal strength could be computed using the following equation:
  (9) $$\begin{array}{c} \begin{array}{c} {{\text{LI}}_{E}|}_{ij}=\frac{E_{C3}^{ij}-E_{C4}^{ij}}{E_{C3}^{ij}+E_{C4}^{ij}} \end{array}. \end{array}$$
(iii) (C3) Calculate ELI over all subjects for four frequency bands using (1) in (10) to (13), where *i* ranges from 1 to 21. To investigate the variation trend of ELI with the parameter *λ*, we vary *λ* in the range of 0 : 0.1 : 1. Specifically, if *λ*=0, only the signal complexity is considered as (8), and besides if *λ*=1, only signal strength is in consideration as (9),
  (10) $$\begin{array}{c} \begin{array}{c} {\text{ELI}|}_{i\delta }=\lambda \cdot {{\text{LI}}_{\text{FE}}|}_{i\delta }+\left(1-\lambda \right)\cdot {{\text{LI}}_{E}|}_{i\delta } \end{array}, \end{array}$$
  (11) $$\begin{array}{c} \begin{array}{c} {\text{ELI}|}_{i\theta }=\lambda \cdot {{\text{LI}}_{\text{FE}}|}_{i\theta }+\left(1-\lambda \right)\cdot {{\text{LI}}_{E}|}_{i\theta } \end{array}, \end{array}$$
  (12) $$\begin{array}{c} \begin{array}{c} {\text{ELI}|}_{i\alpha }=\lambda \cdot {{\text{LI}}_{\text{FE}}|}_{i\alpha }+\left(1-\lambda \right)\cdot {{\text{LI}}_{E}|}_{i\alpha } \end{array}, \end{array}$$
  (13) $$\begin{array}{c} \begin{array}{c} {\text{ELI}|}_{i\beta }=\lambda \cdot {{\text{LI}}_{\text{FE}}|}_{i\beta }+\left(1-\lambda \right)\cdot {{\text{LI}}_{E}|}_{i\beta } \end{array}. \end{array}$$
In summary, PSG data from 21 subjects were studied in this paper. As mentioned before, based on the PSG data quality and other clinical evaluations, 20 seconds C3-A2 and C4-A1 EEG data labelled with normal sleep and OSA were segmented separately for each subject. The EEG decomposition based on the wavelet transform was then performed to acquire the four typical frequency bands. As a result, we got a total of 3360 normal sleep EEG epochs and 3360 OSA EEG epochs as described in Step B1. All the following results were conducted on MATLAB 2018a on a Dell computer with a 3.40 GHz Intel Core i7-2600 CPU and 16.0 GB RAM. This section consists of three main parts: EEG complexity evaluation, EEG strength evaluation, and computation of the enhanced laterality index.

## 3. Results

### 3.1. EEG Complexity Evaluation

To investigate the signal complexity, we computed fuzzy entropy [29] on each epoch of normal sleep and OSA EEGs. The computation procedure was given in Step B1. In this study, we do not intend to investigate the influence of different parameters, thus we just apply the same default parameters for each epoch that *m*=2, *n*=2, and *r* equals 0.2 times of the standard deviation. We present the fuzzy entropy values calculated for all subjects in Table 2, in which the mean value and standard deviation are given. To investigate the statistical properties of fuzzy entropy among different EEG bands, between left and right hemispheres, and between normal sleep and obstructive apnea, the paired samples *T* test was given in Tables 3–5, in which *p* < 0.05 was annotated in bold and with ‘^*∗*^', indicating that significant difference exists. Significant and consistent changes in fuzzy entropy can be seen between 4 frequency bands. It is also interesting to note that differences also exist between C3 and C4 channel or normal sleep and OSA epochs, which is just not that numerically significant.

Based on the signal complexity computed by fuzzy entropy, the hemispheric asymmetry during normal sleep and OSA is evaluated in this section by LI, in which *λ*=1, *Q*_LH_=FE_*c*3_, and *Q*_RH_=FE_*c*4_.  Figure 5 illustrates the LI distributions along with FE_*c*3_ and FE_*c*4_ for four frequency bands. The two axes denote FE_*c*3_ and FE_*c*4_ respectively, and the pixels in each figure indicate the corresponding LI. Concretely, on one hand, if LI scatters in the upper right corner, i.e., FE_*c*3_ is close to 1, whereas FE_*c*4_ is close to 0, we can make the conclusion that the left hemisphere dominates the main brain activity. On the other hand, the main brain activity is concentrated in the right hemisphere if LI locates in the lower left corner. Both (A) and (B) in Figure 5 show clear boundaries among *δ*, *θ*, *α*, and *β* bands. However, the LI distribution in (A) and (B) is also similar, showing a symmetry respect to the diagonal for both normal and obstructive apnea EEG segments, contradicting the existing conclusion of asymmetric sleep in apneic human patients [18, 20]. Consequently, LI performs poorly in distinguishing between normal sleep and OSA just using one representative quantity.

### 3.2. EEG Strength Evaluation

Similar results on EEG strength evaluation are then presented in this section. The computation procedure of EEG epoch strength is given in Step B2. To give a comparable presentation with Figure 5, the computed values of signal strength are normalized between 0 and 1.  Table 6 shows the normalized signal strength of 4 frequency bands calculated for all subjects. To investigate the statistical properties of signal strength among different EEG bands, between left and right hemispheres, and between normal sleep and obstructive apnea, the paired samples *T* test is also given in Tables 7–9, in which *p* > 0.05 was annotated with ‘^*∗*^', indicating that no significant difference exists. According to Table 7, signal strength has significant differences between each other among four frequency bands. Besides, differences in signal strength also exist between C3 and C4 or normal sleep and OSA epochs.

At the same time, LI based on signal strength is calculated to investigate the asymmetry between two hemispheres. The LI distribution is then illustrated in Figure 6. Consistent conclusions could be drawn that strength differences among the 4 bands are significant since the LI distribution boundaries are clear. However, since both (A) and (B) in Figure 6 illustrate symmetry distributions of LI, it seems that LI with only signal strength in consideration is also unable to make the distinction between normal sleep and OSA. The poor performance of LI is further manifested in this section with just signal strength in consideration.

### 3.3. Enhanced Laterality Index

To address the problems of LI mentioned in Sections 3.1 and 3.2, we calculate and present the results in this section based on the proposed ELI. According to (10–13), ELI is computed as the sum of *λ* times of the LI calculated based on the signal complexity and 1 − *λ* times of the LI calculated based on the signal strength.

Figure 7 shows the result of ELI, in which 4 randomly selected subjects are illustrated in subfigures (a) ∼ (d). Each column in Figure 7 shows the ELI values of *δ*, *θ*, *α*, and *β* bands for normal sleep and OSA EEG. Specifically, so as to investigate the influence of parameter *λ*, we vary it in the range of 0 : 0.1 : 1. More precisely, when *λ* is set to 0, only the signal complexity is considered, as presented in Section 3.1, whereas when *λ* is set to 1, only signal strength is in consideration, as presented in Section 3.2. To save space, we only show the ELI results of 4 typical choices of parameter *λ*. In Figure 7, (a1) ∼ (d1) illustrate the results when *λ*=0.2, *λ*=0.4 for (a2) ∼ (d2), *λ*=0.6 for (a3) ∼ (d3), and *λ*=0.8 for (a4) ∼ (d4).

The line graphs in Figures 7(a)–7(d) clearly manifest that there is a significant difference between normal sleep and OSA EEG. The ELI values of OSA EEG are generally higher than those of normal sleep for all 4 frequency bands, and the differences between each other increase gradually with the parameter. In order to give an overall relationship of ELI with each of *δ*, *θ*, *α*, and *β* for all parameter *λ* in [0,1], the average ELI from 21 subjects are computed and presented in Figure 8. It is illustrated that the relationship of ELI and *λ* is linear, which can also be concluded from the definition equation [1]. Besides, it is proven again that ELI in obstructive sleep apnea is always higher than that in normal sleep, and the difference intends to increase with the parameter *λ*.

## 4. Discussion

In the work of this paper, we aim to propose a novel measure for assessing functional asymmetries across frequency bands called the enhanced laterality index (ELI) by taking more than one representative quantity into account simultaneously in investigating the functional differences between two cerebral hemispheres.

### 4.1. The Functional Differences in EEG Frequency Bands

The functional interpretation to various EEG frequency bands has gone through a revolution in recent studies. The low-frequency bands, including *δ*, *θ*, and *α* bands, were believed to ascribe the broad functional role of cortical inhibition to slow rhythms, while the high-frequency bands, i.e., *β* and *γ* bands (30–100 Hz), were associated with cortical activation and neural networks integration [30]. However, other studies have given new claims on the functional interpretations of EEG bands. Stein et al. [31] reported that all bands marked different levels of cortical, top-down integration except the *δ* band. The functional meaning of high-frequency bands was associated with cognitive processing, integration and learning, while low-frequency bands correlated with either working memory engagement or active inhibition of task-irrelevant cortical regions. The functional differences of EEG frequency bands have also been reported in various studies. In the work of analysing language hemispheric lateralization, young adults were reported rightward lateralization in the *δ* frequency band, while all aged groups showed left-lateralized linguistic effects concerning the *β* band [32]. Thus, the *β* band was believed to represent the most reliable EEG marker of language hemispheric asymmetry in children and adults. While in the study of hemispheric lateralization of brain activity during cognitive tasks, Bolduc et al. [33] revealed left prefrontal lateralization on the total spectrum amplitude power and right occipital lateralization in the *δ* band. At the same time, right frontal lateralization in *θ* and *β* bands and right lateralization in occipital *δ* activity were also observed during REM sleep. In the work of analysing OSA hemispheric asymmetry of this paper, the signal complexity and signal strength are investigated on various EEG frequency bands. Significant differences are presented in Tables 2 and 6 among 4 bands. On one hand, the lowest fuzzy entropy, or signal complexity, exists in the *δ* band, whereas the *β* band shows the highest signal complexity. Besides, the *α* band also has a significant complexity increment than *θ*. On the other hand, the *δ* band always has the strongest strength, *α* and *β* bands are similar while the *θ* band is commonly extremely smaller than the other three. Figure 7 reveals that ELI values of OSA patients are generally higher than those of normal subjects among 4 bands.

### 4.2. ELI in Investigating Hemispheric Asymmetry during Sleep

Existing publications have manifested that sleep in obstructive apnea patients is significantly disturbed with frequent apnea and arousal events, and these events would lead to functional asymmetry of the brain [20]. In this paper, we first computed the classical laterality index (LI) with signal complexity and signal strength independently, and then, the proposed ELI was calculated by considering both representative quantities simultaneously. Furthermore, the differences in ELI in four frequency bands were also presented to make a deep understanding of the functional asymmetries among frequency bands. In terms of signal complexity, fuzzy entropy was computed. A significant difference in fuzzy entropy values among 4 frequency bands is presented in Table 2. Conclusions would be drawn that the signal complexity grows with frequency, and the functional complexity of the brain during sleep mainly concentrates in the *β* band. However, when it comes to signal strength, as presented in Table 6, a different result would be reported that the functional strength of the brain during sleep mainly concentrates in the *δ* band. Thus, if we only consider signal complexity in the *β* band while ignoring signal strength in the *δ* band, or vice versa, one-sided or even incorrect results would be inevitable. As shown in Figure 9, when only signal strength of *δ* or signal complexity of *β* is considered, conclusions are contradictory. Furthermore, as illustrated in Figures 5 and 6, both normal sleep and obstructive sleep apnea show an overall symmetry on both hemispheres, and we could not observe obvious differences of LI distribution between each other, contradicting the proven fact. However, ELI solves this problem and shows obvious differences between normal sleep and obstructive sleep apnea that ELI values of obstructive apnea EEG are generally higher than those of normal sleep for all frequency bands, as presented in Figure 7. By contrast, we just took into account of two representative quantities simultaneously in ELI, the distinction in functional asymmetry between normal sleep and obstructive sleep apnea was clearly presented.

### 4.3. Representative Quantities

To reflect the hemispheric asymmetry during specific events, such as EEG-arousal or sleep apnea, various features have been extracted in existing publications. For example, power spectrum, voxels, signal correlations, relative phase, and degree of interdependence have been applied independently in [15, 18, 21]. In this work, we extract two physically direct features, i.e., signal complexity and signal strength, to evaluate the functional asymmetry during normal sleep and obstructive sleep apnea.

In existing publications, signal complexity [34–36] has been widely used in EEG-based signal processing such as EEG classification and disease diagnosis. Reports revealed that EEG signal complexity may contain important information on the neural network architectures in the brain on many scales. Thus, the study in EEG signal complexity would help to learn the neural connectivity of the brain. In addition, signal complexity was also believed to be associated with the ability of attending and adapting to a cognitive task. A study on schizophrenia reported that the patients have a significantly lower EEG signal complexity than that of normal subjects. At the same time, the EEG signal complexity also showed significantly higher interhemispheric and intrahemispheric cross-mutual information values in patients compared with the controls [37]. At the same time, signal strength [38], or signal energy, was also a commonly used feature in existing reports. The energy indicates the strength of the signal as it gives the area under the curve of power at any interval of time. A classification system based on signal strength was developed to classify the ictal and seizure-free EEG signals. EEG signal strength was also reported to be helpful in epileptic seizure detection [39].

### 4.4. Limitations and Future Work

Nevertheless, we should also point out the main limitation of this work. It is preliminarily proved that the proposed ELI performs well in assessing hemispheric asymmetry, but discussions on how to choose optimum values for the *λ* are still missing. Considering that sample size is important in determining the optimum *λ*, we think that a different way to determine the optimum *λ* is to explore the weight of signal complexity and signal strength in assessing lateralization of brain function from a physiological perspective in the future work. Besides, the superiority of ELI was verified by considering only two quantities from EEG data. Other features should be carefully extracted and selected from not only EEG data but also fMRI in the future. Since ELI is able to deal with multiple quantities, we believe it will perform better with more representative quantities. In addition, the way of information fusion between different representative quantities is also worth further study and improvement.

## 5. Conclusions

We proposed a novel measure for investigating the functional differences between two cerebral hemispheres called the enhanced laterality index (ELI). Its reliability is manifested by comparison with a traditional laterality index (LI). Compared with existing measures, ELI is theoretically reliable because it would take more than one representative quantity into account when evaluating hemispheric dominances. This is believable because both cerebral hemispheres always have complicated information communications between each other during brain activities. Thus just one kind of quantity is hard to make a comprehensive understanding to the whole brain activity. However, all existing measures merely consider one quantity in this issue, and this is where ELI intend to address. The superiority of ELI is further verified in the experiment for normal sleep and obstructive sleep apnea. Clinical EEG data from 21 OSA patients are involved in this study. Two commonly used features, i.e., signal complexity and signal strength, are extracted from C3-A2 and C4-A1 EEG channels to calculate ELI. Concretely, the signal complexity is evaluated by fuzzy entropy, and the signal strength is evaluated by calculating signal energy. Finally, by comparison with the traditional LI, we present that the ELI is indeed superior in assessing the functional differences of both hemispheres. The future work will be focused on investigating more representative quantities from EEG/fMRI data and improving the way of information fusion.

## Figures and Tables

**Figure 1:** Illustration of 20 s epoch C3-A2 and C4-A1 EEG signals for normal sleep and OSA.

**Figure 2:** PSG signals and event annotations, in which the red box indicates the exact OSA event annotation.

**Figure 3:** (a) Butterworth filter magnitude response, the cutoff frequency is 50 Hz. (b) The frequency spectrum based on the Fourier transform of the original EEG data and the filtered data.

**Figure 4:** Typical frequency bands decomposed from original EEG data based on the wavelet transform. (a) *δ* (1–3 Hz), (b) *θ* (4–7 Hz), (c) *α* (8–13 Hz), and (d) *β* (14–30 Hz).

**Figure 5:** LI distribution along with FE_*C*3_ and FE_*C*4_. Total epochs were presented in (a) normal sleep and in (b) obstructive sleep apnea.

**Figure 6:** LI distribution along with *E*_*C*3_ and *E*_*C*4_. Total epochs were presented in (a) normal sleep and in (b) obstructive sleep apnea.

**Figure 7:** ELI computed with signal complexity and signal strength in consideration. 4 randomly selected subjects are illustrated in subfigures (a)–(d). *λ*=0.2 in (a1) ∼ (d1), *λ*=0.4 in (a2) ∼ (d2), *λ*=0.6 in (a3) ∼ (d3), and *λ*=0.8 in (a4) ∼ (d4).

**Figure 8:** Average ELI from 21 subjects for each of *δ*, *θ*, *α*, and *β*.

**Figure 9:** ELI*|*_*β*+*δ*_ when signal strength of *δ* and signal complexity of *β* are considered simultaneously.

**Table 1:** Demographic details of the subjects studied.

No.	Age	Sex	Sleep efficiency (%)	AHI	Arousal (/h)	SpO_2_ (%)
1	76	M	35.6	16.7	17.4	96
2	64	F	73.0	—	8.2	—
3	51	M	94.3	43.3	19.4	95
4	51	M	—	3.7	—	97
5	18	M	—	37.6	—	94
6	45	F	77.6	—	8.4	—
7	26	M	98.5	70	51.5	93
8	21	M	95.8	35.4	9.1	96
9	53	M	96.8	69.1	43.7	95
10	35	M	91.7	76.6	12.7	91
11	46	F	96.3	3.9	5.4	97
12	51	F	92.1	9.8	3.9	98
13	60	F	91.9	14.0	0.9	97
14	44	M	92.5	31.5	13.8	96
15	85	F	26.2	39.4	7.9	96
16	47	M	87.0	29.7	25.1	97
17	63	F	81.0	30.7	12.5	94
18	44	M	90.1	37.1	15.0	95
19	56	F	—	4.1	—	97
20	34	M	97.1	51.0	23.4	96
21	40	F	84.0	72.3	9.9	98

**Table 2:** Differences in signal complexity for normal sleep and OSA EEG epochs.

Bands	Normal sleep		Obstructive apnea	
	FE_*C*3_	FE_*C*4_	FE_*C*3_	FE_*C*4_
*δ*	0.1412 ± 0.0705	0.1499 ± 0.0749	0.1491 ± 0.0756	0.1547 ± 0.0774
*θ*	0.3473 ± 0.0857	0.3427 ± 0.0972	0.3436 ± 0.0869	0.3483 ± 0.0887
*α*	0.5036 ± 0.0715	0.4940 ± 0.0934	0.4948 ± 0.0733	0.4931 ± 0.0878
*β*	0.6007 ± 0.0776	0.6019 ± 0.1005	0.5859 ± 0.0701	0.5899 ± 0.0769

Mean value and standard deviations are presented for each frequency band. The functional complexity of the brain during sleep mainly concentrates in the *β* band.

**Table 3:** Paired samples *T* test of fuzzy entropy between paired EEG bands.

Bands	Normal sleep		Obstructive apnea	
	FE_C3_	FE_C4_	FE_C3_	FE_C4_
*δ*-*θ*	0.000^*∗*^	0.003^*∗*^	0.000^*∗*^	0.035^*∗*^
*δ*-*α*	0.015^*∗*^	0.004^*∗*^	0.000^*∗*^	0.009^*∗*^
*δ*-*β*	0.000^*∗*^	0.023^*∗*^	0.002^*∗*^	0.011^*∗*^
*θ*-*α*	0.032^*∗*^	0.000^*∗*^	0.043^*∗*^	0.009^*∗*^
*θ*-*β*	0.000^*∗*^	0.009^*∗*^	0.029^*∗*^	0.028^*∗*^
*α*-*β*	0.000^*∗*^	0.008^*∗*^	0.000^*∗*^	0.000^*∗*^

There are significant differences in fuzzy entropy between each pair of frequency bands, whether in normal sleep or obstructive sleep apnea. The asterisks in Table 3 mean that P < 0.05 in the paired samples T test, indicating that significant differences in fuzzy entropy exist between paired EEG bands.

**Table 4:** Paired samples *T* test of fuzzy entropy between two hemispheres.

Bands	Normal sleep	Obstructive apnea
	FE_C3_ - FE_C4_	FE_C3_ - FE_C4_
*δ*	0.004^*∗*^	0.017^*∗*^
*θ*	0.051	0.038^*∗*^
*α*	0.000^*∗*^	0.022^*∗*^
*β*	0.391	0.000^*∗*^

In normal sleep, significant differences in fuzzy entropy between C3 and C4 channels exist in both *δ* and *α* bands, while not in *θ* and *β*. In contrast, significant differences exist in all bands in OSA sleep. The asterisks in Table 4 mean that P < 0.05 in the paired samples T test, indicating that significant differences in fuzzy entropy exist between two hemispheres.

**Table 5:** Paired samples *T* test of fuzzy entropy between normal sleep and obstructive apnea.

Bands	**F** **E**_**C**3_	**F** **E**_**C**4_
	Normal sleep-obstructive apnea	Normal sleep-obstructive apnea
*δ*	0.001^*∗*^	0.123
*θ*	0.556	0.001^*∗*^
*α*	0.000^*∗*^	0.190
*β*	0.026^*∗*^	0.000^*∗*^

In the C3 channel, significant differences in fuzzy entropy between normal sleep and OSA sleep exist in *δ*, *α*, and *β*. While in the C4 channel, significant differences exist in *θ* and *β*. The asterisks in Table 5 mean that P < 0.05 in the paired samples T test, indicating that significant differences in fuzzy entropy exist between normal sleep and obstructive apnea.

**Table 6:** Difference in signal strength for normal sleep and OSA EEG epochs.

Bands	Normal sleep		Obstructive apnea	
	*E*_*C*3_	*E*_*C*4_	*E*_*C*3_	*E*_*C*4_
*δ*	0.6919 ± 0.0917	0.6863 ± 0.0943	0.6853 ± 0.0862	0.6874 ± 0.0915
*θ*	0.1218 ± 0.0643	0.1316 ± 0.0674	0.1283 ± 0.0680	0.1302 ± 0.0670
*α*	0.5504 ± 0.0649	0.5400 ± 0.0760	0.5450 ± 0.0643	0.5433 ± 0.0685
*β*	0.4159 ± 0.0725	0.4075 ± 0.0771	0.4147 ± 0.0743	0.4095 ± 0.0706

Mean value and standard deviations are presented for each frequency band. The functional strength of the brain during sleep mainly concentrates in the *δ* band.

**Table 7:** Paired samples *T* test of signal strength between paired EEG bands.

Bands	Normal sleep		Obstructive apnea	
	*E*_*C*3_	*E*_*C*4_	*E*_*C*3_	*E*_*C*4_
*δ*-*θ*	0.024^*∗*^	0.006^*∗*^	0.000^*∗*^	0.045^*∗*^
*δ*-*α*	0.005^*∗*^	0.026^*∗*^	0.031^*∗*^	0.007^*∗*^
*δ*-*β*	0.002^*∗*^	0.003^*∗*^	0.042^*∗*^	0.013^*∗*^
*θ*-*α*	0.000^*∗*^	0.000^*∗*^	0.033^*∗*^	0.008^*∗*^
*θ*-*β*	0.000^*∗*^	0.001^*∗*^	0.024^*∗*^	0.030^*∗*^
*α*-*β*	0.018^*∗*^	0.004^*∗*^	0.000^*∗*^	0.002^*∗*^

There are significant differences in signal strength between each pair of frequency bands, whether in normal sleep or obstructive sleep apnea. The asterisks in Table 7 mean that P < 0.05 in the paired samples T test, indicating that significant differences in signal strength exist between paired EEG bands.

**Table 8:** Paired samples *T* test of signal strength between two hemispheres.

Bands	Normal sleep	Obstructive apnea
	*E*_*C*3_ –*E*_*C*4_	*E*_*C*3_ –*E*_*C*4_
*δ*	0.085	0.083
*θ*	0.005^*∗*^	0.163
*α*	0.000^*∗*^	0.396
*β*	0.021^*∗*^	0.006^*∗*^

In normal sleep, significant differences in signal strength between C3 and C4 channels exist in *θ*, *α*, and *β* bands, while not in *δ*. In contrast, significant differences exist in all bands in OSA sleep. The asterisks in Table 8 mean that P < 0.05 in the paired samples T test, indicating that significant differences in signal strength exist between two hemispheres.

**Table 9:** Paired samples *T* test of signal strength between normal sleep and obstructive apnea.

Bands	*E*_*C*3_	*E*_*C*4_
	Normal sleep-obstructive apnea	Normal sleep-obstructive apnea
*δ*	0.006^*∗*^	0.486
*θ*	0.026^*∗*^	0.308
*α*	0.004^*∗*^	0.010^*∗*^
*β*	0.614	0.054

In the C3 channel, significant differences in signal strength between normal sleep and OSA sleep exist in *δ*, *α*, and *β*. While in the C4 channel, significant differences exist in *θ* and *β*. The asterisks in Table 9 mean that P < 0.05 in the paired samples T test, indicating that significant differences in signal strength exist between normal sleep and obstructive apnea.

## Data Availability

The polysolmnography data used to support the findings of this study have not been made available because the data are restricted by the Sleep Medical Centre of Shandong Provincial Hospital, China, in order to protect patient privacy. Data are available from the corresponding author for researchers who meet the criteria for access to confidential data.
